The article "Analysis of Risk Factors of Coal Chemical Enterprises Based on Text Mining" was published in 2023. Journal: J Environ Public Health.

# Analysis of Risk Factors of Coal Chemical Enterprises Based on Text Mining

**DOI:** 10.1155/2023/4181159

**Published:** 2023-01-28

**Authors:** Zheng Li, Min Yao, Zhenmin Luo, Xinping Wang, Qianrui Huang, Chang Su

**Affiliations:** ^1^College of Safety Science and Engineering, Xi'an University of Science and Technology, Xi'an 710054, China; ^2^Institute of Management Science, Ningxia University, Yinchuan 750021, China; ^3^College of Management, Xi'an University of Science and Technology, Xi'an 710054, China

## Abstract

Coal chemical enterprises have many risk factors, and the causes of accidents are complex. The traditional risk assessment methods rely on expert experience and previous literature to determine the causes of accidents, which has the problems such as lack of objectivity and low interpretation ability. Analyzing the accident report helps to identify typical accident risk factors and determines the accident evolution rule. However, experts usually judge this work manually, which is subjective and time-consuming. This paper developed an improved approach to identify safety risk factors from a volume of coal chemical accident reports using text mining (TM) technology. Firstly, the accident report was preprocessed, and the Term Frequency Inverse Document Frequency (TF-IDF) was used for feature extraction. Then, the *K*-means algorithm and apriori algorithm were developed to cluster and for the association rule analysis of the vectorized documents in the TF-IDF matrix, respectively to quickly identify the hidden risk factors and the relationship between risk factors in the accident report and to propose targeted safety management measures. Using the sample data of 505 accidents in a large coal chemical enterprise in Western China in the past seven years, the enterprise accident reports were analyzed by text clustering analysis and association rule analysis methods. Through the analysis, six accident clusters and 13 association rules were obtained, and the main risk factors of each accident cluster were further mined, and the corresponding management suggestions were put forward for the enterprise. This method provides a new idea for coal chemical enterprises to make safety management decisions and helps to prevent safety accidents.

## 1. Introduction

The COVID-19 epidemic has severely affected the energy markets [1]. China has turned its attention to coal in order to ensure national energy security again. In 2020, coal accounted for about 56.8% of China's primary energy consumption, which is still the leading energy in China [2]. As a necessary form of vital energy in China and an important organic raw material, coal is widely used in cooking, chemical fertilizer production, rubber, plastics, and other coal chemical industries [3, 4]. The coal chemical industry takes coal as the raw material, then converts coal into gas, liquid, solid fuel, and chemicals through chemical processing, and then produces various chemical products. Developing the coal chemical industry is essential to promote clean and efficient coal utilization and to ensure national energy security [5].

There are over 100 large-scale coal chemical enterprises worldwide, with nearly 400 modern gasifiers. In comparison, there are more than 3000 coal chemical production enterprises in China with more than 1 million employees in the coal chemical industry [6]. Developing a safe, green, and environmentally friendly coal chemical industry can effectively supplement China's oil and gas resources shortage. However, there were many problems, such as serious waste of resources and insufficient attention to safety and environmental protection [7]. Most of the production processes of the coal chemical industry have harsh process conditions and complex production devices. A safety accident in a coal chemical enterprise may cause significant harm to personnel, equipment, facilities, and the environment [8]. In addition, during the average production of coal chemical enterprises, the continuous operation time is generally long, the work intensity is high, and the staff is prone to negligence, leading to safety accidents.

The safety production situation of China's chemical industry is still grim and complex. From 2016 to 2019, 784 chemical accidents in China caused 1002 deaths. From January to November 2021, 127 domestic chemical accidents resulted in 157 deaths. Therefore, it has become an urgent problem for many scholars to accurately identify the potential safety hazards of coal chemical enterprises [9].

Common safety accidents in coal chemical enterprises mainly include fire, explosion, and leakage of toxic gas or liquid [10]. Most of the accidents originated from process areas, storage areas, and waste storage or disposal areas. The direct causes of chemical accidents mainly include mechanical failure, human errors, and violent reactions, of which human errors account for the most significant proportion [11]. The commonly used safety assessment methods in coal chemical enterprises are diversified, and the qualitative methods include preliminary hazard analysis, safety checklist, HAZOP analysis, and FMEA analysis. Quantitative evaluation methods include the Dow Chemical method and probabilistic risk assessment. Approaches that combine qualitative and quantitative methods include safety checklist, event tree, and accident tree [6].

However, safety risk identification in those models was limited to experience-based methods (e.g., literature review and questionnaires). Various accident causation theories and models were proposed based on the induction analysis of accidents, such as the Swiss cheese model, the man-made disaster theory, and the System-Theoretic Accident Model and Processes (STAMP). [12]. These theories have highlighted the primary mechanisms of how risk factors might cause an accident. However, the accident causal model does not clearly define detailed safety risk factors. That is mainly because most studies take expert experience and previous literature, as the primary source in determining the causes of accidents, resulting in a lack of objectivity and low interpretation ability. Secondly, when studying the causal relationship of accident causes, researchers often put forward assumptions and variable combinations through observation or related theories, lacking an objective basis [13]. Using the data mining method to deeply mine disaster information gives the excellent value for accident prevention.

Although the industrial fields differ, the accidents have similar trajectories [14]. Learning from accidents is a pivotal link to preventing future injuries [15], focusing on determining the event's root cause [16]. As explicit knowledge, the text information in accident reports is easy to share [17], and hundreds of accident reports can form a valuable knowledge database. The accident report has an outstanding value in understanding the details of the accident sequence, including important text information related to corrective and preventive maintenance after the accident [18]. Analyzing the accident report helps to identify typical accident risk factors and determine the accident's cause, type, location, and severity [19]. Currently, this work mainly depends on the judgment of experts in the field, which is subjective and time-consuming [20]. In particular, enterprises have accumulated many safety accident reports and hidden danger troubleshooting reports. These reports are presented in unstructured text, which increases the difficulty of quickly and accurately identifying risk factors from many text datasets.

In recent years, data analysis in accident investigation reports has provided a new way to study the causes of accidents [21]. Through extensive research of accident reports, text mining can better understand the causes of accidents and significantly improve the accuracy of accident prediction [22]. In the field of chemical safety management, work on anomaly detection [23], ontology-based knowledge acquisition [24], and process alarm prediction [25] have been undertaken based on accident texts. Despite such work, no existing method meets the demands of both universality and accuracy, and there is still no efficient, convenient universal tool for extracting risk factors from coal chemical accident cases.

This paper is data-driven and theory-driven for better prevention and control of the potential safety hazards of coal chemical enterprises and to ensure safe production. It proposes a text mining method to automatically identify the critical risk factors hidden in the accident report, which can help enterprises find valuable information and implicit knowledge. A specific dictionary in the field of the coal chemical industry is established, which plays a vital role in the text mining workflow. Six accident clusters are obtained through text cluster analysis, and the accident causes of these accident clusters are found, and improvement measures are put forward. Through the association rule analysis of the excavated risk factors, 13 association rules are obtained. According to these association rules, targeted security management can be carried out.

The chapters are arranged as follows. The background of text mining and related works is presented in Section 2.  Section 3 includes the details of the proposed approach.  Section 4 introduces the case application of this method in a large coal chemical enterprise in Western China.  Section 5 is the summary of this study.

## 2. Literature Review

The production process conditions of the coal chemical industry are harsh, and the production equipment is complex. Scholars have carried out much risk research in the coal chemical industry. In order to improve the risk management and control ability of coal chemical enterprises, Miao studied the dynamic risk management and control model of coal chemical enterprises and developed the corresponding application software [26]. Chen introduced the modeling method and management strategy of the domino effect and pointed out future research directions and challenges to better protect the chemical industry from the impact of catastrophic accidents [11]. Zhang established a quantitative relationship between probability and equipment damage degree and developed a reliability probability model related to specific types of chemical processing equipment [27]. Shahriar studied the risk of oil and gas pipeline leakage accidents through the sustainability assessment method and used bow tie analysis based on fuzzy theory to prevent significant accidents [28]. Although these studies have improved the risk assessment method for the coal chemical process, risk management still faces substantial challenges. Major coal chemical accidents are low-frequency events; the traditional risk assessment methods that rely on coal chemical accident data cannot be effectively applied to production practice [29].

With the rapid development of science and technology such as artificial intelligence, 5G, big data, the Internet of things, and cloud platform, more data are available than ever. The international data group predicts that data will increase from 33 billion TB in 2018 to 175 billion TB in 2025 [30]. In addition, most of these data are in unstructured formats, including audio, video, and free text. Unstructured data accounts for about 80%. Knowledge can be found from various information sources, while the text is still the largest existing information source.

Information overload, that is, the amount of data generated, has exceeded its processing and analysis capacity. It is a growing concern in many industries, especially a large number of free-text data extracted under human supervision. Henke believes that 76% of work activities need natural language understanding. Therefore, developing automated methods to deal with natural language texts effectively are essential [31].

Text mining, also known as knowledge discovering in texts (KDT), processes a large number of unstructured text data through natural language processing (NLP) technology to obtain new knowledge and valuable information [32]. In the 1950s, Luhn first proposed applying the idea of word frequency statistics to automatic classification, creating a precedent in the research and application of text mining [33]. The concept of “text mining“ was first proposed by Feldman in the paper First International Conference on Text Mining and Knowledge Discovery [34].

Text mining is a branch of data mining and covers many research fields. As we all know, data mining can mine the seemingly scarce potential knowledge in massive explosive data. When the mined data appears in text, this mining method can be called text mining. Because the information hidden in the report is unstructured, the computer cannot process it, while manual text processing is time-consuming and error-prone. Through text preprocessing and feature extraction in text mining technology, text information can be scientifically abstracted and transformed into a mathematical model that the computer can recognize. Of course, the theories and methods of machine learning, information processing, pattern recognition, statistics, computer linguistics, and other disciplines need to be used in this process [35]. Text data have the characteristics of large volume, diversity, velocity, low-value density, and the 4V feature of big data [36]. Compared with the wide application of machine learning in image processing, speech recognition, and other fields, text data mining is challenging.

Text mining is becoming a new research hotspot and has been widely used in many fields, such as medicine, commerce, and security. The most famous application in the medical field is PubGene, a search engine containing many life science and biomedical data. It can visually show the possible relationship between keywords and literature data. In the business field, enterprises use text mining technology's intelligent web crawler function to collect information about the market, competitors, and market environment related to enterprises and further analyze this information to adjust the enterprise development strategy [37]. In the safety field, many scholars use text mining technology to analyze coal mines, rail transit, ship collision, aviation, and other accidents, extract the causes of accidents, and then put forward practical safety management suggestions. For example, Lin developed a text mining method based on keyword extraction and topic modeling to identify the key concerns and dynamics of on-site inspection problems of construction projects to make decisions better [38]. Sarkar developed a text-mining-based prediction model by using fault tree analysis (FTA), and Bayesian network (BN) could predict the occurrence of accidents attributable to different primary causes [39]. Raviv used text mining and *K*-means cluster analysis of 212 crane-related accident reports to find that technical failure is the most dangerous risk factor [40]. Hughes introduced a semiautomatic technology for classifying text-based short-distance call reports in the GB railway industry to type many unstructured texts [41]. Singh identified the nine most common accident paths and the corresponding prevention strategies through text mining (workplace observation and high-risk control plan) and reactivity data (event records) [42].

The techniques used in text mining include information extraction, topic tracking, text classification, text clustering, association analysis, information visualization, latent semantic analysis, and emotion analysis [37].

Text clustering is essential in data mining and machine learning [43]. The purpose is to find helpful knowledge or patterns from unstructured or semistructured text sets [44]. Given a document set, we need to divide the documents into several clusters so that the documents in the same cluster are similar. Unlike classification methods, clustering is a typical unsupervised learning method [45], and we do not need to label documents in advance. Therefore, text clustering technology can be considered when there is no annotation information of documents. Text clustering has a wide range of applications, such as topic detection and tracking [46], document summary [47], and search results clustering [48]. A wealth of techniques has been proposed for text clustering, including spectral methods [49], matrix factorization [50], hierarchical methods [51], partitional approaches [52], and model-based methods [53], in addition to further approaches based on semantic similarity [54], evolutionary algorithms [55] and concept factorization [56].

According to the accident causation theory, accidents cannot be caused by one factor but by breaking through the bottom line of the defense system under the joint action of different factors. In order to further reveal the patterns between different factors, association analysis needs to be carried out to extract strong association rules between risk factors. Association rule mining is an essential branch of data mining technology. Agrawal first proposed the concept of association rule mining, the association or correlation between itemsets in the database, which is also known as shopping basket analysis [57]. The well-known algorithms like apriori [57], FP-growth [58], and ECLAT [59] and their derivatives have introduced efficient frequent itemset mining processes for association rules. Other types of itemsets mining methods have been introduced for rule mining, such as approximate [60], rare [61], and uncertain itemset mining [62]. These mined itemsets have been used to produce several forms of rules like multilevel and multidimensional association rules.

Given the subjectivity of traditional risk factor analysis methods in the field of the coal chemical industry, this paper combines data-driven and theory-driven. It proposes a method and process of text mining, which can objectively extract risk factors from many accident case data.

## 3. Methodology

This paper presents the process and method of extracting risk factors from accident reports based on text mining, as shown in Figure 1. In the safety management process, coal chemical enterprises have accumulated many accident reports, hidden danger troubleshooting records, and other text data, and constituted a knowledge treasure waiting for in-depth excavation. After preprocessing and feature extraction of the content of a large number of informants, it is transformed into a structured dataset. The text clustering and association rule analysis are carried out. Finally, combined with the mined tacit knowledge, the daily safety management decision-making of the enterprise is carried out.

### 3.1. Text Preprocessing

Text preprocessing is the fundamental link of text mining, which aims to clean and standardize the corpus. It usually includes screening steps, removing stop words, word segmentation, and part-of-speech tagging. Chinese text preprocessing does not need stem analysis, citation, and case normalization, which makes text preprocessing different from English text. Four substeps are designed: data screening, removing stop words, constructing a domain dictionary, and word segmentation.

1. *Data Screening*. Because of the randomness of text data records and many professional terms and idioms, text normalization is required before Chinese word segmentation, which is usually completed by regular expressions [63]. This study takes the accident report as the initial database. Sincethe preparation of accident reports has corresponding requirements and the text is relatively standardized, this paper only needs to delete duplicate and defective reports (for example, incomplete reports) during data screening.
2. *Removing Stop Words*. Stop words refer to words and punctuation marks that frequently appear in the text but have no functional meaning and are not helpful to the analysis of the theme of the text content. These meaningless words can be deleted by importing the stop words list. The stop words list can be found and downloaded from the Modern Chinese Function Words Dictionary in the Google and Baidu input methods.
3. *Constructing Domain Dictionary*. Due to the diversity of human language, there are significant differences in the description of security risk factors. In order to better segment text, it is necessary to construct a customized domain dictionary in advance. The existing dictionary construction methods are mainly corpus-based, knowledge-based, and combinations [64].
4. *Word Segmentation*. By locating the term boundary, the corpus is decomposed into discrete and linguistically meaningful terms [65]. Chinese word segmentation recombines continuous Chinese sentences into word sequences according to specific rules. By removing stop words, eliminating the interference of meaningless words, and further introducing the constructed domain dictionary, word segmentation can be carried out directly.

### 3.2. Feature Selection

After text preprocessing and feature vectorization, the feature dimension of the text is still very high. In order to reduce the computational complexity, feature extraction is needed. Feature extraction is a dimensionality reduction method that calculates a feature's score value according to a feature evaluation function, sorts these features according to the score results, and selects features with high score values as feature items. It reduces the number of features and the computational complexity of modeling and improves clustering performance.

As a traditional feature selection method, the Term Frequency Inverse Document Frequency (TF-IDF) is usually used as a feature evaluation function for feature extraction [66]. The TF-IDF matrix has been widely used to train shallow learning models [67], such as SVM, KNN, and NB. The TF of keywords is expressed as

(1) $$\begin{array}{c} tf_{i,j}=\frac{n_{i,j}}{\sum_{K}n_{k,j}}\text{,} \end{array}$$

where *n*_*i*,*j*_ denotes the number of occurrences of the keyword *t*_*i*_ that appears in the accident record document *d*_*j*_ and ∑_*K*_*n*_*k*,*j*_ is the number of all keywords in the accident record document *d*_*j*_.

The IDF of keywords is expressed as

(2) $$\begin{array}{c} i\;df_{i}=\log\frac{\left|D\right|}{1+\left|\left\{j:t_{i}\in d_{j}\right\}\right|}\text{,} \end{array}$$

where |*D*| represents the total number of accident record documents and |{*j* : *t*_*i*_ ∈ *d*_*j*_}| is the number of documents containing keyword *t*_*i*_ to avoid this item being zero and the divisor being zero, and it is generally expressed as 1+|{*j* : *t*_*i*_ ∈ *d*_*j*_}|. IDF means that the fewer times a keyword appears in an accident record document, the greater the weight given to the keyword. It is the opposite of TF's idea, but it is susceptible to rare keywords.

TF-IDF combines the advantages of TF and IDF [68], indicating that the weight of a keyword will increase with the number of times it appears in an accident record document and decrease with the number of relevant accident records in the database:

(3) $$\begin{array}{c} TF-IDF_{i,j}=tf_{i,j}\times i\;df_{i}\text{.} \end{array}$$

Using the TF-IDF method to calculate the weight of the keywords obtained from word segmentation, we can identify the important keywords within the document and realize feature extraction. It can effectively reduce many worthless words and improve the performance of subsequent clustering analysis and the effect of correlation analysis.

### 3.3. Text Clustering Analysis

The textual documents usually need to be classified according to content similarity [69]. For small datasets, we can manually classify text into specific clusters. However, clustering a large number of documents will be very time-consuming. Therefore, it is crucial to develop accurate and fast methods in text mining [70].

*K*-means clustering is the most commonly used clustering technology [71]. This algorithm can be extended to large datasets and applied in many applications [72]. *K*-means clustering algorithm takes the sum of squares errors (SSEs) as the objective function to minimize the SSEs between texts in *K* clusters. The cluster center *e*_*i*_ of cluster *E*_*i*_ can be expressed as

(4) $$\begin{array}{c} e_{i}=\frac{1}{n_{i}}\underset{n\in E_{i}}{\sum }x\text{.} \end{array}$$

The SSE between texts is calculated as follows:

(5) $$\begin{array}{c} SSE=\overset{K}{\underset{i=1}{\sum }}\underset{n\in E_{i}}{\sum }\cos\;{\left(e_{i},x\right)}^{2}\text{,} \end{array}$$

where *x* represents the text object, *E*_*i*_ is the *i*^th^ cluster, *n*_*i*_ denotes the number of samples therein, and *e*_*i*_ is the center of cluster *E*_*i*_.

With *K*-mean clustering, the vectorized documents in the TF-IDF matrix are divided into *K* distinct clusters based on Euclidean distance to the centroid of a cluster [73].

Firstly, the cluster value *K* needs to be given, and then the centroid position is recalculated after all eigenvalues are assigned to the nearest centroid. This process is repeated until convergence occurs, and no further changes occur [74]. The initially set *K* value directly affects the clustering effect. Rousseeuw proposed the silhouette coefficient method that provides a graphic display to evaluate the cluster quality and judge the text clustering effect [75]. Assuming that the original data are divided into *K* clusters, for each vector *i* in the cluster, give *a*(*i*) as the average distance from vector *i* to other vectors in the same cluster, indicating the degree of cohesion in the cluster and *b*(*i*) as the average distance from vector *i* to all vectors in the nearest cluster, indicating the degree of separation between clusters. *S*(*i*) is the silhouette coefficient of vector *i*, which can be expressed as

(6) $$\begin{array}{c} S\left(i\right)=\frac{b\left(i\right)-a\left(i\right)}{\max\;\left\{a\left(i\right),b\left(i\right)\right\}}\text{.} \end{array}$$

Averaging the silhouette coefficients of all vectors is the contour coefficient of the cluster. The value range of the contour coefficient is [−1, 1], 1 indicates high-density clustering, −1 indicates incorrect classification, and the value around 0 indicates overlapping clusters.

### 3.4. Association Rule Analysis

There are many algorithms for mining association rules, among which the most classic algorithm is the apriori algorithm [76]. The basic idea of the apriori algorithm is to find the frequent itemset according to the set support until the frequent *K *+* *1 itemset do not exist. Corresponding to the general steps of the association rule algorithm in data mining, text association analysis also includes two stages: (1) aearching frequent itemsets and (2) generate association rules based on frequent itemsets.

Three methods are widely used in the literature to evaluate the quality of association rules: support, confidence, and lift.

The expression of support (*S*) is

(7) $$\begin{array}{c} S=\left(X\Rightarrow Y\right)=P\left(X\cup Y\right)\text{.} \end{array}$$

In the formula, *P* represents the probability that both itemsets *X* and *Y* co-occur in a transaction. Moreover, the support is symmetrical; that is, the support of *X*⇒*Y* is equivalent to the support of *Y*⇒*X*.

The expression of confidence (*C*) is

(8) $$\begin{array}{c} C=\left(X\Rightarrow Y\right)=P\left(Y\left|X\right.\right)=\frac{P\left(X\cup Y\right)}{P\left(X\right)}\text{.} \end{array}$$

This formula represents the conditional probability of event Y under the condition that event X occurs. It is not symmetric; the confidence of the rule *X*⇒*Y* may be different from the confidence of the rule *Y*⇒*X*.

Support and confidence are probability values, and their value interval is [0, 1]. The closer the value is to 1, the stronger the relationship between events.

The expression of lift (*L*) is

(9) $$\begin{array}{c} L\left(X\Rightarrow Y\right)=\frac{Confi\;de\;nce}{P\left(Y\right)}=\frac{P\left(Y\left|X\right.\right)}{P\left(Y\right)}=\frac{P\left(X\cup Y\right)}{P\left(X\right)P\left(Y\right)}\text{.} \end{array}$$

The lift is the conditional probability of itemset *Y* when itemset *X* in the transaction set is divided by the probability of itemset *Y* in the transaction set occurring alone. Generally, the lift value is compared with 1, less than 1 indicates a negative correlation between the antecedent and consequent items, greater than 1 indicates a positive correlation between the two, and equal to 1 indicates no correlation.

## 4. Case Application

This section will introduce the case application. We investigated a large coal chemical enterprise in Western China and obtained 505 accident reports from 2015 to 2020. The accident reports record the department, name, time, grade, nature, injury degree, and process of the accident. This paper chose Python language to mine and analyzed the obtained text database.

### 4.1. Text Preprocessing

The integrity and standardization of the obtained accident reports were checked. It was found that 505 accident reports were filled in a standardized format and completed in content, which can be analyzed in the next step.

Combined with Modern Chinese Function Words, Baidu, and Harbin Institute of technology's stop-words list, a Chinese stop-words list containing 1893 words, such as punctuation and function words is sorted out. The meaningless words in the accident report were deleted by importing the stop-words list.

This study used the combination method based on corpus and knowledge to construct a dictionary in the coal chemical industry. The specialized dictionary comes from safety engineering, chemical engineering, and risk management. At the same time, enterprise safety managers were invited to sort out some professional words with industry recognition combined with the expression characteristics of accident reports. These two parts of vocabulary constitute the domain dictionary used in this study.

The widely used Jieba Chinese word segmentation toolkit was installed in anaconda. Word segmentation and part-of-speech tagging were carried out on text data combined with the established domain dictionary. However, the words obtained through word segmentation cannot be mined and analyzed directly. On the one hand, too many keywords contain unhelpful interference items, leading to dimensional disaster. On the other hand, the obtained keywords only have frequency statistics, and a simple word frequency cannot reflect the importance of vocabulary.

### 4.2. Feature Extraction

Scikit learn is a machine learning software package based on Python, which constructs a feature matrix for the obtained keywords by calling the countvectorizer function. The TF-IDF vectorizer is called to calculate the weight of each feature according to the TF-IDF algorithm (see Table 1).

In this paper, the keywords that occur more than three times are regarded as high-frequency words, and the TF-IDF values of keywords are arranged in the descending order, and the top 10% are defined as feature items. It can be seen from the above table that the weight value of each feature item is relatively small because the weight value is related to the frequency of the word in the document, and the entire database contains thousands of words. The weight value of the feature item is only a relative value, which plays a role in ranking the importance. The feature items with higher weight values mainly include gasifier, central control room, coke oven gas, interlock, pressure, and induced draft fan, indicating that the accidents are mostly related to the above feature items. By comparing the accident records, it was found that the shutdown and maintenance accidents are caused by the failure of equipment components such as gasifier, induced draft fan, compressor, reactor, and pipeline rupture. Interlocking accidents are caused by excessive fluctuation of process parameters such as flow, pressure, liquid level, and temperature. The feature items with high weight can accurately reflect the relevant information about frequent accidents. Cluster analysis and association rules require further analysis of detailed accident characteristics and causes.

### 4.3. Text Clustering Analysis

The last section calculated the weight of the extracted feature items and constructed a spatial vector model. This section will calculate the similarity between documents for text clustering analysis.

The silhouette coefficient combines the cohesion and separation of clustering to evaluate the effect of clustering. Use the silhouette score function to determine the *K* value of cluster analysis. The result is shown in Figure 2. When the *K* value is 6, the silhouette coefficient is the largest, close to 1, indicating that high-density clustering can be obtained.

*K*-means cluster analysis is carried out on 505 accident reports, and six clusters are finally obtained, as shown in Figure 3, see Table 2 for detailed results.

The accident reports included in the six clusters are 121, 105, 87, 82, 71, and 39. The leading causes of accident clustering can be found by summarizing the feature items, as shown in Table 3. Cluster 0 contains the most accidents, mainly personal injury accidents. The causes of the accidents include insufficient safety awareness of employees, failure to take protective measures, nonstandard operation, misoperation, and untimely communication, reflecting the lack of employees' occupational safety knowledge and safety awareness. Cluster 1 mainly refers to equipment and parts damage accidents. The causes of the accidents include induced draft fan parts damage, motor damage, and compressor parts damage, indicating that enterprises need to strengthen the inspection and maintenance of the frequently above faulty equipment. Cluster 2 mainly refers to leakage accidents. The causes of accidents include economizer leakage, pipeline blockage/rupture, and flange leakage, reflecting the need for enterprises to formulate and improve regular inspection systems and assessment mechanisms. Cluster 3 mainly refers to production line shutdown accidents caused by large fluctuations in process parameters such as flow, liquid level, and pressure, which indicates that enterprises should strengthen the training of employees on the operation skills of Distributed Control System and Safety Monitoring System and formulate emergency plans for various emergencies. The leading causes of the accidents in Cluster 4 are that the sundries on the equipment and site are not cleaned in time, resulting in equipment tripping, fire, and other accidents, indicating that the cleanliness of the enterprise is insufficient. Cluster 5 mainly refers to traffic accidents in the plant area. The causes of the accidents are insufficient safety awareness of employees and failure to comply with traffic rules. It is also necessary to strengthen the safety training of employees and formulate regulations on traffic travel in the plant area.

### 4.4. Association Rule Analysis

According to the data format required by the association rules, the Boolean matrix was constructed using the feature items in the accident report, as shown in Table 4.

Each column represents an item; the accident cause item is mined from the text. Each line represents a transaction, i.e., accident report *D*_*i*_. 1 indicates that the cause of the accident appears in the accident report, and 0 means that it does not. Set the minimum support threshold to 0.1 and the minimum confidence threshold to 0.3. Search frequent sets and filter out the rules with a lift greater than 1 to obtain 13 association rules, as shown in Table 5.

The reason for the relatively low support of these rules is that the vocabulary contained in the database is very large, and the dimension of the feature matrix is too high, so the frequency of the two feature items appearing together is low. However, the confidence of these association rules is almost greater than 0.5, which means that the feature items in the rules have a strong correlation. It can be seen from the above table that 38.5% of the association rules obtained are related to the central control, indicating that in case of abnormal conditions in the daily production process, the central control will issue operation instructions in the shortest time to avoid worse results. Abnormal flow, load, and liquid level fluctuations will lead to abnormal process pressure changes. The disturbance of load will also cause the abnormality of pressure, flow, motor, and other equipment parameters. The probability of compressor failure and unqualified propylene products appearing together in the accident reports is 14.2%, and the probability of unqualified propylene products caused by compressor failure is 56.7%. The lifting degree of the circulating pump and reactor is 8.203, indicating that they have a very significant positive correlation.

The lifting value of the final 13 rules is greater than 1, indicating that the consequent item of the rules is greatly affected by the antecedent item. According to association rules, the obtained rules have obvious practical significance and can carry out targeted safety management.

### 4.5. Results of Practical Application

According to the text clustering results and the characteristics of departments and posts, the case enterprise has designed different knowledge question banks and randomly selected questions every month to test the employees. Employees can access the question bank through mobile phones any time for learning. At the same time, the enterprise focused on the inspection and maintenance of induced draft fan, motor, compressor, economizer, and other equipment prone to frequent failures for two months. According to the correlation analysis results, the enterprise has added the linkage monitoring function of essential process parameters in the central control system to prevent domino events caused by excessive fluctuations of process parameters. Through statistical analysis of accident reports in 2021, it is found that the number of accidents decreased by 16.9% year-on-year, of which human factor accidents, equipment failure accidents, and interlocking accidents decreased by 18.4%, 11.1%, and 14.3%, respectively, and the safety situation of the enterprise was significantly improved.

## 5. Conclusion

To accurately identify the risk factors in coal chemical enterprises and effectively prevent safety accidents, this paper developed an improved approach to identify safety risk factors from a volume of coal chemical accident reports using TM technology.

Firstly, the features of the preprocessed accident text are extracted using the TF-IDF method. Secondly, based on the characteristics of coal chemical enterprises, the K-means algorithm and apriori algorithm are developed to perform clustering and association rule analysis on the feature matrix, respectively. The analysis results identify the main risk factors of accident clustering and the correlation between risk factors. Finally, the method is applied to a large chemical enterprise in Western China, and six accident clusters and 13 association rules are obtained. The main risk factors of each accident cluster are further analyzed, and the corresponding safety management measures are proposed. The final results show that the method proposed in this paper can quickly identify the critical risk factors hidden in the accident report, and their relationships and help enterprises to carry out scientific management and decision-making.

In the future, more enterprise data should be selected to verify the method. At the same time, it is necessary to summarize the accident types and causes in more detail to identify better the risk factors existing in the enterprise.

## Figures and Tables

**Figure 1:** Text mining process of accident reports in the coal chemical industry.

**Figure 2:** Silhouette coefficient of accident text clustering.

**Figure 3:** Visual results of accident text clustering analysis.

**Table 1:** Feature item weight value (top 30).

No.	Feature item	Weight
1	Gasifier	0.1053
2	Central control room	0.0954
3	Coke oven gas	0.0795
4	Interlocking	0.0729
5	Coke quenching vehicle	0.0648
6	Pressure	0.0640
7	Liquid level	0.0623
8	Load	0.0601
9	Induced draft fan	0.0589
10	Coking plant	0.0542
11	Compressor	0.0532
12	Vibration	0.0504
13	Temperature	0.0518
14	Flow	0.0472
15	Reactor	0.0441
16	Pipeline	0.0437
17	Speed of revolution	0.0426
18	High-pressure cylinder	0.0424
19	Shut down	0.0399
20	Pure benzene	0.0399
21	Feed pump	0.0377
22	Slag lock bucket	0.0376
23	Boiler	0.0355
24	Electric machinery	0.0355
25	Coking plant	0.0349
26	Lean solution pump	0.0349
27	Valve	0.0331
28	Surge	0.0330
29	Trip	0.0322
30	Overhaul	0.0320

**Table 2:** Clustering results of accident reports.

Cluster no.	Accident record content	Word segmentation
0	At about 14 : 00 on October 19, 2015, when operators polished the pipe orifice at the DN600 short joint of circulating water near the primary cooler of coking plant 2#, the splash prevention measures were not standardized. The sparks fell on the insulation cotton attached with tar, industrial naphthalene, and other carbon compounds, resulting in smoke and fire. After the fire was founded, the construction personnel and operators quickly used fire extinguishers to put the open fire on-site and reported to relevant leaders in time.	Coking plant, primary cooler, circulating water, polish, fire prevention measures, nonstandard, mars, tar, industrial naphthalene, carbonaceous compound, insulation cotton, smoke, catch fire, and fire extinguisher
1	At 22 : 39 on February 19, 2016, 4# boiler an induced draft fan tripped, the DCS panel reported the failure of the thin oil station, and the lubricating oil pressure dropped to 0. Through inspection by site personnel, it was found that the upper end of the electric heating contactor of the induced draft fan was heated and burned out, its power air switch tripped, and the power switch of the control cabinet of the thin oil station tripped. At 23 : 16, after cutting off the electric heating power supply and turning on the control cabinet's power switch, the induced draft fan of party a usually starts, and the 4# boiler restores the load.	Induced draft fan, trip, thin oil station, fault, lubricating oil, pressure, decline, electric heating contactor, heating, burn out, power switch, control cabinet, and load
2	At 6 : 15 on August 30, 2017, 5# boiler working condition was abnormal, and the deviation between main steam flow and feedwater flow was 100 t/h. After inspecting and confirming economizer leakage, it was reported to the general dispatcher to apply for boiler shutdown. After boiler shutdown, the 72nd and 76th low temperature economizers from east to west were leaked, and the leaking pipes were intercepted and discharged.	Working condition, abnormal, steam, flow, deviation, economizer, leakage, shutdown, low temperature, pipeline
3	At 22 : 38 on July 29, 2018, the membrane recovery compressor PDT-3514 gave a low-pressure alarm, and the low alarm value was 135kpa. The oil pump G-370 A/B double pumps started, and the pressure of membrane recovery compressor C-351 did not return to normal, so it was immediately interlocked and shut down.	Membrane recovery, compressor, low voltage alarm, oil pump, interlocking, and shutdown
4	At 16 : 40 on February 28, 2017, pulverized coal flow in the 1# pulverized coal pipeline of 1# gasifier suddenly dropped to 0. The gasification workshop analyzed and judged that there were sundries in the angle valve. After reporting to the plant leaders, it decided to dismantle and inspect the 1# pulverized coal angle valve, and some bag fragments were found in the angle valve.	Gasifier, pulverized coal, pipeline, flow, reduce, central control, main operation, angle valve, shutdown, fragment, and purge
5	At about 23 : 20 on June 16, 2016, Xu, the first shift operator of the gasification workshop of the methanol plant, collided with an electric vehicle travelling in the opposite direction about 300 meters in front of the gate of the chemical base on his way to work, resulting in the rupture of Xu's left eyeball. He is now sent to the branch of the hospital for treatment.	Methanol plant, gasification workshop, operator, reverse driving, electric vehicle, collide, and fracture
…	…	…

**Table 3:** Accident cause analysis.

Clustering	Feature item	Main accident causes
0	Maintenance, violation, blind plate, nonstandard, protective measures, fire, smoke, disassembly, cleaning, safety rope, slip, fall, high temperature, scald, crush, respirator, and fainting	Lack of safety awareness, failure to take protective measures, nonstandard operation, misoperation, and untimely communication
1	Induced draft fan, motor, circuit board, bearing, compressor, switch, damage, fault, over temperature, burn out, trip, shutdown	Equipment failure, induced draft fan parts damage, motor damage, compressor parts damage, over temperature, and switch trip
2	Low temperature and high temperature economizer, flange, boiler, pipeline, water wall, leakage, rupture, leakage point, water level, rise, furnace, pressure, shutdown, and maintenance	Economizer leakage, pipeline rupture, water wall rupture, flange leakage, and pipeline blockage
3	Coke oven gas, flow, parameters, alarm, temperature, vibration, water level, abnormality, pressure, liquid level, low and rise fluctuation, interlocking, overrun, and too high and too fast shutdown	The gas flow/liquid level/pressure/temperature fluctuates wildly, and the vibration amplitude is too large
4	Angle valve, pulverized coal, gasifier, quench chamber, blockage, sundries, material accumulation, trip, and shutdown	Sundries are not cleaned on time
5	Carelessness, vehicle, collision, knockdown, fracture, bus, and injury	Lack of safety awareness and failure to comply with traffic rules

**Table 4:** The Boolean matrix used by association rules.

	Pressure	Flow	…	Load	Speed of revolution
*D *_1_	1	0	…	1	0
*D *_2_	1	1	…	0	1
*D *_3_	0	1	…	1	1
…	…	…	…	…	…
*D *_484_	0	0	…	1	0

**Table 5:** Association rules for accident causes.

Rules	Support	Confidence	Lift
flow ⇒ central control	0.107	0.396	1.875
central control ⇒ scene	0.198	0.842	1.749
central control ⇒ pressure	0.136	0.579	2.132
interlocking ⇒ central control	0.112	0.553	2.616
pipeline ⇒ central control	0.124	0.667	2.842
flow ⇒ pressure	0.158	0.584	2.101
load ⇒ pressure	0.160	0.546	1.962
load ⇒ flow	0.155	0.527	1.953
load ⇒ electric machinery	0.147	0.364	2.519
compressor ⇒ propylene	0.131	0.567	2.667
liquid level ⇒ pressure	0.194	0.600	2.133
circulating pump ⇒ reactor	0.131	0.769	8.203
pipeline ⇒ compressor	0.142	0.525	2.665

## Data Availability

The data used to support the findings of this study are available from the corresponding author upon request.
